# Analysis of the Clinical Effect of Visual Electrophysiological Examination Combined with Targeted Health Education Nursing in Children

This article has been retracted.

**DOI:** 10.1155/2023/3543790

**Published:** 2023-04-11

**Authors:** Yanan Qiu, Lan Xiong

**Affiliations:** Department of Ophthalmology, Lanzhou University Second Hospital, Lanzhou, Gansu 730000, China

## Abstract

**Objective:**

To analyze the clinical effect of visual electrophysiological examination combined with targeted health education nursing in children.

**Methods:**

A total of 100 children who underwent visual electrophysiological examinations in the Ophthalmology Department of our hospital from March 2019 to March 2021 were selected as the study subjects. The children were randomly divided into two groups, the control group and the observation group, with 50 children in each group. Children in the control group received routine nursing, while those in the observation group received a combination of routine nursing and targeted health education nursing. The nursing satisfaction, degree of cooperation with examination, examination time, changes in the psychological state, and the stress response of the children and their families were then compared and analyzed.

**Results:**

The nursing satisfaction of the observation group was higher than that of the control group (94.0% vs. 80.0%) (*P* < 0.05). The degree to which children in the observation group cooperated with examination was higher than that of children in the control group (96.0% vs. 78.0%) (*P* < 0.05). The average time spent on VEP and ERG examinations by children in the observation group was 6.33 ± 1.37 hours and 55.25 ± 4.92 hours, respectively, significantly lower than that of 12.45 ± 1.02 hours and 70.36 ± 5.31 hours, respectively, spent by children in the control group (*P* < 0.05). After intervention, the depression, hostility, anxiety, and obsession scores of children in the observation group were all significantly lower than those of children in the control group (*P* < 0.05). There was an increase in the heart rate, respiratory rate, and mean arterial pressure in children from both groups, but the magnitude of increase in the observation group was much smaller than that in the control group (*P* < 0.05).

**Conclusion:**

The combination of visual electrophysiological examination and targeted health education nursing in children has a remarkable clinical effect. It improves the children's degree of comfort as well as the parents' degree of satisfaction. It also reduces the time spent on examinations, facilitates the smooth completion of examinations, and improves the efficiency of examinations. This nursing method is one that merits more widespread promotion and clinical application.

## 1. Introduction

In recent years, due to the popularization of electronic products and the increase of academic pressure, the prevalence of myopia in children in China has been increasing year by year, and it has shown a younger trend [1]. Additionally, the development of myopia increases the risk of retinal detachment, macular choroidopathy, and other blinding eye diseases. In addition, because the current society still has high requirements for good distance vision, myopia is not only harmful to children's personal physical and mental health but also detrimental to social development and talent training. Therefore, the prevention and control of children's myopia is immensely critical [2, 3].

The increased level of attention that human beings pay to ophthalmic disorders has led to continuous developments in visual electrophysiological technology [4, 5]. Visual electrophysiological examination is a noninvasive, objective, and quantitative examination method that can reflect the dysfunction of the visual system from the retina to the visual center. It has good application value in disease diagnosis, condition monitoring, prognosis, and judgment of curative effect, and it is also a good objective examination method to study the visual function of DME. At present, optical coherence tomography and visual electrophysiological examination have been widely used in the diagnosis and prognosis of DME [6, 7]. This technology has now become one of the most important functional examinations in the field of ophthalmology [8]. There are 3 main components of the examination, namely, electroretinogram (ERG), electrooculogram (EOG), and visual evoked potential (VEP), all of which are objective and noninvasive [9, 10]. It has proved to be of great value in the detection of declining visual function and is now widely used in the diagnosis, differentiation, prognosis, and pathogenesis of various ophthalmic disorders [11, 12].

Children present a special challenge because they are not as attentive and cooperative as adults. On the one hand, children in this age group are often afraid of hospitals and medical staff, and on the other hand, their comprehension and cooperation abilities are poor. Also, their families do not have a good understanding of visual electrophysiological examination, which often leads to psychological issues and longer times spent on examination. This tends to affect the authenticity of the results [13]. High-quality nursing is a nursing model following the concept of people-oriented on the basis of routine nursing. Traditional health education emphasizes form and ignores content, and it is easy to ignore the participation factor of children, which not only wastes time but also is not conducive to knowledge mastery. Therefore, this study adopts targeted health education with targeted strategies.

Therefore, targeted health education for patients undergoing visual electrophysiological examination can not only improve parents' understanding of the procedure but can also help them get rid of any concerns that they might have. It can also reduce the incidence of adverse reactions and ensure successful completion of the examination.

## 2. Materials and Methods

### 2.1. Clinical Information

A total of 100 children who underwent visual electrophysiological examinations in the Ophthalmology Department of our hospital from March 2019 to March 2021 were selected as the study subjects. The children were randomly divided into two groups, the control group and the observation group, with 50 children in each group. The control group consisted of 26 males and 24 females, aged between and 6 and 12 years, with an average age of 8.26 ± 1.38 years. The observation group consisted of 25 males and 25 females, aged between 6 and 13 years, with an average age of 8.39 ± 1.51 years. There was no significant difference in the baseline data of children in the two groups (*P* > 0.05), and the data were comparable.

The randomization was carried out using an online web-based randomization tool (freely available at https://www.randomizer.org/). For concealment of allocation, the randomization procedure and assignment were managed by an independent research assistant who was not involved in screening or evaluation of the participants.

The original sample size calculation estimated that 50 patients in each group would be needed to detect a 3-point difference between groups in a 2-sided significance test with a power of 0.8 and an alpha error level of 0.05.

The trial was done in accordance with standards of Good Clinical Practice and the Declaration of Helsinki. The trial protocol and all amendments were approved by the appropriate ethics body at each participating institution (KI-LI20100505). All patients provided written informed consent before enrolment. The trial protocol has been published online and is available with the full text of this article.

Inclusion criteria included the following:

1. Children who did not undergo other eye surgeries or medical therapies during the study period.
2. Children with complete clinical data.

Children and their parents were informed of the study, and the parents signed the informed consent form.

### 2.2. Examination Method

The RETI-Port 21 Compact of the German ROLAND ophthalmic electrophysiological diagnostic system was used. The electrodes were placed according to the manufacturer's instructions.

*VEP Examination*. The active electrode was placed 1.5–2.0 cm above the occipital tubercle, the reference electrode was placed in the middle of the forehead, and the ground electrode was placed on the earlobe.

*ERG Examination*. 1 drop of Benoxi eye solution was placed in the conjunctival sac. The corneal contact lens electrode was then placed 5 minutes later. The reference electrode was placed on the lateral aspect of both eyes, and the ground electrode was placed on the earlobe.

### 2.3. Nursing Method

The routine nursing method was adopted for children in the control group. Before the examination, family members of the children were informed of the precautions. During the examination, they assisted in fixing the child's head and paying attention to the child's situation. After the examination, they were again informed of other necessary precautions [14]. Targeted health education and nursing (similar to the one described for children in the control group) were adopted for children in the observation group. Before the examination, nursing staff provided a detailed explanation of visual electrophysiological examination and a brief explanation of the procedure to the children and their parents [15]. This was done to help them have a basic understanding of the examinations, some circumstances that may arise during the examination, and how to avert them. Children and their parents were asked to voice out their concerns, and the nursing staff provided appropriate explanations to dispel these concerns. This was done in order to increase their level of trust in the medical staff and to improve the child's cooperation. The child was accompanied throughout the examination process. Local anesthetics were administered to relieve physiological factors such as tears and visual fatigue that can otherwise affect the examination [16, 17]. After ERG examination, the nursing staff rinsed the conjunctival sac with normal saline, applied eye drops to prevent infection, and instructed the child to refrain from rubbing the eyes. Children who underwent VEP examination were advised to avoid long-term exposure to bright light for 6–8 hours and to wear sunglasses when travelling. Upon discharge, children and their parents were given the necessary guidance and were instructed to seek medical attention immediately if they had any problems.

### 2.4. Observational Indicators

1. Nursing satisfaction: A nursing satisfaction survey was carried out using a questionnaire developed by the hospital. The highest possible score is 100. A score of 25 or less is unsatisfactory, that above 25 but not greater than 75 is relatively satisfactory, and that greater than 75 is satisfactory. The higher the score, the higher the nursing satisfaction.
2. Degree of cooperation with the examination: An individual was said to have highly cooperated with the examination if the individual was cooperative throughout the examination, without being very emotional or nervous, and the examination did not have to be stopped mid-way. The degree of cooperation was said to be good if the individual was mildly stressed, but the examination proceeded regardless. Lastly, an individual was said to have a low degree of cooperation with the examination if the individual was not cooperative throughout the examination process and struggled physically, necessitating an interruption in the examination process.
3. Time spent on examination.
4. Psychological state: The psychological state of the two groups of children was assessed before and after intervention using the self-rating symptom scale (SCL-90) based on 4 aspects: depression, hostility, anxiety, and obsession. Each aspect was scored from 1 to 5, and the result was interpreted as “none, mild, moderate, or severe.” The lower the score, the better the psychological state.
5. Stress response: The stress response indices of the two groups of children were assessed and compared. These included the heart rate, respiratory rate, and mean arterial pressure.

### 2.5. Statistical Methods

If the parameter beta is either a difference of means, a log odds ratio, or a log hazard ratio, then it is reasonable to assume that *b* is unbiased and normally distributed.

SPSS22.0 was used to process the data. The enumeration data (*n* (%)) and measurement data (±*s*) were subjected to chi-square and *t* tests, respectively. *P* < 0.05 was considered statistically significant.

## 3. Results

### 3.1. Clinical Information

There was no significant difference in the clinical information between children from the two groups (*P* > 0.05) (Table 1).

### 3.2. Nursing Satisfaction

The nursing satisfaction of the observation group (94.0%) was significantly higher than that of the control group (80.0%) (*P* < 0.05) (Table 2).

### 3.3. Degree of Cooperation with Examination

The degree of cooperation with examination in the observation group (96.0%) was significantly higher than that in the control group (78.0%) (*P* < 0.05) (Table 3).

### 3.4. Time Spent on Examination

The average time spent on VEP and ERG examinations by children in the observation group was 6.33 ± 1.37 hours and 55.25 ± 4.92 hours, respectively, significantly lower than that of 12.45 ± 1.02 hours and 70.36 ± 5.31 hours, respectively, spent by children in the control group (*P* < 0.05) (Table 4).

### 3.5. Psychological State

Before intervention, there was no significant difference in the depression, hostility, anxiety, and obsession scores of children in the two groups. However, after intervention, the depression, hostility, anxiety, and obsession scores of children in the observation group were all significantly lower than those of children in the control group (*P* < 0.05) (Table 5).

### 3.6. Stress Indicators

Before intervention, there was no significant difference in the heart rate, respiratory rate, and mean arterial pressure between children from the two groups. After intervention, there was an increase in the heart rate, respiratory rate, and mean arterial pressure in children from both groups, but the magnitude of increase in the observation group was much smaller than that in the control group (*P* < 0.05) (Table 6).

## 4. Discussion

The development of the visual system is immature at birth, and after being stimulated by normal visual experience, the shape and function of the visual pathway gradually develop to perfection. In this process, the best corrected visual acuity of one eye or both eyes caused by abnormal visual experience for various reasons is lower than normal. Amblyopia will seriously affect the development of children's visual function, which will become obstacles in their future education, employment, and work, thus affecting their life development [18, 19]. With the improvement of living standards and the enhancement of people's health awareness, more and more parents realize the importance of children's eye health, so more and more children with amblyopia are diagnosed. The purpose of amblyopia treatment is to eliminate visual inhibition, improve vision, and restore binocular vision. The earlier the treatment is started, the better the treatment effect is. The best treatment period is 3 to 5 years old, yet children in this age group are often afraid of hospitals and medical staff on the one hand and have poor understanding and cooperation skills on the other hand [20, 21]. Targeted health education nursing has become a very popular nursing model in recent years. It can provide patients with targeted nursing interventions at both the physical and psychological levels [22, 23].

In this study, targeted health education and nursing were adopted for children undergoing visual electrophysiological examinations. Differences in ways of thinking, personalities, and receptive abilities that naturally exist between children and their family members were taken into consideration before carrying out targeted health education. This greatly improved parents' understanding of the examination and improved the children's cooperation and compliance to the examination [24, 25]. Because ERG must be performed in a dark room, some children may be afraid of the dark environment. Therefore, it is important to let the children familiarize themselves with the environment before the examination begins. Thereafter, depending on how the child reacted to the dark environment, appropriate encouragement and communication can be offered to relieve the child's tension and anxiety. The pupil must be dilated before an ERG examination can be performed. It is important that precautions that must be taken after pupillary dilation are explained to the child in advance. After the surface anesthetic has been applied onto conjunctival sac, the corneal contact lens electrode must be placed carefully, patiently, and correctly. While this is being done, the examiner must take the initiative to ask the child if there is any discomfort. During the examination, the child should be told to fixate his or her gaze on the optotype to avoid affecting the quality of the image acquired. After the examination, it is important to look out for signs of corneal damage such as redness, photophobia, and tearing. After 24 hours, the child (or the parents) must be called and asked about any signs of discomfort that the child may be having. This is done to ensure that children undergoing visual electrophysiological examinations are cared for throughout the process.

The results of this study showed that the nursing satisfaction of the observation group was significantly higher than that of the control group. At the same time, the degree of cooperation with examination in the observation group was significantly higher than that in the control group. The average time spent on VEP and ERG examinations by children in the observation group was significantly lower than that spent by children in the control group. These findings suggest that targeted health education nursing can improve cooperation among the subjects, facilitate the smooth completion of examinations, and reduce the time spent on examinations. Poor cooperation among subjects stems from psychological factors, mainly the unfamiliar environment, lack of trust in the examiner, and lack of relevant knowledge concerning the examination. This also reflects that most of the children have a certain fear of hospitals and medical staff; on the other hand, children at this age have poor understanding and cooperation ability and low treatment compliance.

In this study, children in the observation group and their family members received a background introduction of the examiner and detailed information concerning the examination procedure in advance. Before the examination, huge emphasis was placed on psychological guidance of the examinee. The examination room was kept clean, neat, and tidy, and the examinee was made familiar with the environment. This cleared any psychological barriers that the examinee may have harbored prior to the examination. The examinee was accompanied throughout the examination process to prevent him or her from developing negative emotions that can otherwise result in him or her not cooperating with the examination altogether. The results of this study showed that the depression, hostility, anxiety, and obsession scores of children in both groups decreased after intervention, but the decrease was more pronounced in the observation group than in the control group.

The results of this study also showed that there was an increase in the heart rate, respiratory rate, and mean arterial pressure in children from both groups, but the magnitude of increase in the observation group was much smaller than that in the control group. This shows that the use of targeted health education and nursing in visual electrophysiological examination can help to fully understand the subject's psychological status and concerns and provide the necessary guidance and education [26, 27]. This goes a long way in reducing such feelings as depression, hostility, anxiety, and obsession and ensuring the smooth progress of examinations and the authenticity of results. Furthermore, it reduces the time spent on examinations [28–30]. To establish a good interpersonal relationship between high-quality psychological care and children, it is necessary to communicate in their own way and take into account the feelings of the children. This also allows children to avoid the fear of back room testing. Targeted health education can more accurately point to the knowledge blind spots of rehospitalized patients through good early evaluation and solve the actual problems of patients from the perspective of children. However, individuals have different personalities, and individualized and targeted self-management education should be given at any time as needed, with particular attention paid to the physical and psychological education and counseling of preschool children, school-age children, and adolescents [31, 32].

Although this study has certain guiding significance, there are some limitations. This study only included children from a single center. This research conducted eye health education on campus and found that most young people lacked knowledge about eye health, neglected routine eye examinations, and did not pay attention to eye hygiene. In the early stage of the experiment, some students were skeptical or even resistant to the TCM therapy. Through publicity and explanation, on-site demonstration, and evaluation of efficacy after treatment, it gradually gained more attention and recognition from students and parents.

## 5. Conclusion

The combination of visual electrophysiological examination and targeted health education nursing in children has a remarkable clinical effect. It improves the children's degree of comfort as well as the parents' degree of satisfaction. It also reduces the time spent on examinations, facilitates the smooth completion of examinations, and improves the efficiency of examinations. This nursing method is one that merits more widespread promotion and clinical application.

## Figures and Tables

**Table 1:** Comparison of clinical information.

Group	Control group (*n* = 50)	Observation group (*n* = 50)	*t*/*x*^2^	*P*
Sex			0.04	0.841
M/F	26/24	25/25		
Age			0.449	0.654
Range	6∼12	6∼13		
Average age	8.26 ± 1.38	8.39 ± 1.51		
Ocular disease			0.041	0.839
High-degree myopia	20	21		
Pseudoblindness	3	2		
Color anomalopia	4	4		
Retinal detachment	6	5		
Retrobulbar neuritis	4	6		
Strabismus	5	4		
Fundus disease	3	5		
Ametropic amblyopia	4	3		

**Table 2:** Comparison of nursing satisfaction (*n*, %).

Group	*n*	Satisfied	Relatively satisfied	Unsatisfied	Total degree of satisfaction (%)
Observation group	50	27	20	3	47 (94.0%)
Control group	50	14	26	10	40 (80.0%)
*X* ^*2*^					4.332
*P*					0.037

**Table 3:** Comparison of degree of cooperation (*n*, %).

Group	*n*	Highly cooperative	Relatively cooperative	Uncooperative	Total degree of cooperation (%)
Observation group	50	26	22	2	48 (96.0%)
Control group	50	11	28	11	39 (78.0%)
*X* ^*2*^					29.936
*P*					<0.001

**Table 4:** Comparison of time spent on examination ($\bar{x}$ ± *s*).

Group	*n*	VEP examination time (h)	ERG examination time (h)
Observation group	50	6.33 ± 1.37	55.25 ± 4.92
Control group	50	12.45 ± 1.02	70.36 ± 5.31
*T*		25.336	14.76
*P*		<0.001	<0.001

**Table 5:** Comparison of psychological state between the two groups before and after intervention ($\bar{x}$ ± *s*).

Group	*n*	Depression		Hostility		Anxiety		Obsession	
		Before intervention	After intervention	Before intervention	After intervention	Before intervention	After intervention	Before intervention	After intervention
Observation group	50	2.16 ± 0.31	0.72 ± 0.17	2.26 ± 0.38	0.77 ± 0.15	2.33 ± 0.27	0.71 ± 0.15	2.15 ± 0.36	0.70 ± 0.23
Control group	50	2.17 ± 0.32	1.47 ± 0.24	2.23 ± 0.39	1.42 ± 0.18	2.32 ± 0.28	1.34 ± 0.13	2.18 ± 0.37	1.25 ± 0.14
*X* ^*2*^		0.778	7.264	0.961	6.847	0.668	5.784	0.914	4.367
*P*		0.194	<0.001	0.327	<0.001	0.128	<0.001	0.277	<0.001

**Table 6:** Comparison of stress indicators between the two groups before and after intervention ($\bar{x}$ ± *s*).

Group	*n*	HR (beats/min)		RR (breaths/min)		MAP (mmHg)	
		Before intervention	After intervention	Before intervention	After intervention	Before intervention	After intervention
Observation group	50	73.57 ± 8.38	80.71 ± 6.14	21.28 ± 2.11	24.08 ± 2.93	80.52 ± 7.18	83.08 ± 6.62
Control group	50	73.69 ± 8.42	89.63 ± 9.38	21.94 ± 2.12	28.84 ± 3.19	80.33 ± 7.20	89.53 ± 6.96
*X* ^*2*^		0.071	5.626	1.56	7.771	0.132	4.748
*P*		0.944	<0.001	0.122	<0.001	0.895	<0.001

## Data Availability

All data generated or analyzed during this study are included in this article.

## References

[1] Zhou J., Dai H., Zhang Y. (2022). Differences in contrast sensitivity between children with amblyopia and normal children. *Chinese Journal of Optometry and Vision Science*.

[2] Wang X., Xing X., Wang S. (2022). Atropine suppression therapy and occlusion therapy in the treatment of children with anisometropic amblyopia. *International Journal of Ophthalmology*.

[3] Xiao L., Zhang H., Li S. (2022). Status and influencing factors of amblyopia in preschool children in Zigong City, Sichuan Province. *South China Journal of Preventive Medicine*.

[4] Almeida L. F. B., Kattah M., Ventura L. O. (2021). Pattern-reversal visual evoked potential in children with congenital zika syndrome. *Journal of Pediatric Ophthalmology and Strabismus*.

[5] Ameri H., Naser M., Choudhury F., Rao N. A. (2021). Electroretinogram and visual field correlation in birdshot chorioretinopathy. *Asia-Pacific Journal of Ophthalmology*.

[6] Zhang L., Li L., Zhou X., Xia F., Zhang Z. (2013). Visual electrophysiological examination in diagnosis of hepatic encephalopathy. *World Journal of Neuroscience*.

[7] Yin Z. Q., Tao Z., Li S. Y. (2020). Paying attention to the standardization of visual electrophysiological examination. *Chinese Journal of Ophthalmology*.

[8] Brouwer A. H., Wit G. C., ten Dam N. H., Wijnhoven R., Genderen M. M., Boer J. H. (2020). Electroretinogram abnormalities in non-infectious uveitis often persist. *Acta Ophthalmologica*.

[9] Carrarini C., Russo M., Pagliaccio G. (2021). Visual evoked potential abnormalities in dementia with Lewy bodies. *Neurophysiologie Clinique*.

[10] Ciuffreda K. J., Yadav N. K., Ludlam D. P. (2017). Binasal occlusion (BNO), visual motion sensitivity (VMS), and the visually-evoked potential (VEP) in mild traumatic brain injury and traumatic brain injury (mTBI/TBI). *Brain Sciences*.

[11] Covey T. J., Golan D., Doniger G. M. (2021). Visual evoked potential latency predicts cognitive function in people with multiple sclerosis. *Journal of Neurology*.

[12] Creel D. J. (2019). Electroretinograms. *Handbook of Clinical Neurology*.

[13] Creel D. J. (2019). Visually evoked potentials. *Handbook of Clinical Neurology*.

[14] Sarossy M., Crowston J., Kumar D., Weymouth A., Wu Z. (2021). Prediction of glaucoma severity using parameters from the electroretinogram. *Scientific Reports*.

[15] Shuffrey L. C., Rodriguez C., Rodriguez D. J. (2021). Delayed maturation of P2 flash visual evoked potential (VEP) latency in newborns of gestational diabetic mothers. *Early Human Development*.

[16] Tekavčič Pompe M., Šuštar M. (2019). Flicker electroretinogram recorded with portable ERG device in prematurely born schoolchildren with and without ROP. *Documenta Ophthalmologica*.

[17] Terracciano R., Sanginario A., Barbero S., Putignano D., Canavese L., Demarchi D. (2020). Pattern-reversal visual evoked potential on smart glasses. *IEEE Journal of Biomedical and Health Informatics*.

[18] Zhang X., Hu L. (2022). Research progress on non-visual impairment of children with amblyopia. *China Journal of Traditional Chinese Medicine*.

[19] Wang P., Yang Y., Zhang B. (2022). Effects of visual perception training based on binocular push-pull model on visual perception, binocular accommodation and visual acuity in 3-6-year-old children with myopia and amblyopia. *Chinese Journal of Integrative Traditional Chinese and Western Medicine*.

[20] Jing L., Shi J., Tan X. (2022). Clinical study of macular retinal thickness in children with hyperopia anisometropic amblyopia before and after treatment. *International Journal of Ophthalmology*.

[21] Wang Z., Li N., Cao S. (2022). Research on the status quo of life quality and its influencing factors in children with amblyopia. *International Journal of Ophthalmology*.

[22] Creel D. J. (2019). The electrooculogram. *Handbook of Clinical Neurology*.

[23] Dai D. K., Yang L., Meng H. H., Chen X. P., Tao L. Y. (2021). Characteristics of visual evoked potential in different parts of visual impairment. *Fa Yi Xue Za Zhi*.

[24] Dmitriev A. V., Dmitriev A. A., Linsenmeier R. A. (2021). K^+^-dependent Müller cell-generated components of the electroretinogram. *Visual Neuroscience*.

[25] Dziadkowiak E., Sebastian A., Wieczorek M. (2021). Visual evoked potentials as potential biomarkers of visual function in patients with primary sjögren’s syndrome. *Journal of Clinical Medicine*.

[26] Ekayanti M. S., Mahama C. N., Ngantung D. J. (2021). Normative values of visual evoked potential in adults. *Indian Journal of Ophthalmology*.

[27] Hébert M., Mérette C., Gagné A. M. (2020). The electroretinogram may differentiate schizophrenia from bipolar disorder. *Biological Psychiatry*.

[28] Miyagishima K. J., Zhang C., Malechka V. V., Bharti K., Li W. (2020). Direct-coupled electroretinogram (DC-ERG) for recording the light-evoked electrical responses of the mouse retinal pigment epithelium. *Journal of Visualized Experiments: JoVE*.

[29] Nadolski N. J., Wong C. X. L., Hocking J. C. (2021). Electroretinogram analysis of zebrafish retinal function across development. *Documenta Ophthalmologica*.

[30] Nittmann M. G., Aher A. J., Kremers J., Tzekov R. (2021). Relationship between stimulus size and different components of the electroretinogram (ERG) elicited by flashed stimuli. *Documenta Ophthalmologica*.

[31] Strong J., Lattof S. R., Maliqi B., Yaqub N. (2021). Experiences of private sector quality care amongst mothers, newborns, and children in low- and middle-income countries: a systematic review. *BMC Health Services Research*.

[32] Gelkop C., Kagan I., Rozani V. (2021). Are emotional intelligence and compassion associated with nursing safety and quality care? A cross-sectional investigation in pediatric settings. *Journal of Pediatric Nursing*.

